# Comparative Analysis of Skin Cancer (Benign vs. Malignant) Detection Using Convolutional Neural Networks

**DOI:** 10.1155/2021/5895156

**Published:** 2021-12-11

**Authors:** Mohammed Rakeibul Hasan, Mohammed Ishraaf Fatemi, Mohammad Monirujjaman Khan, Manjit Kaur, Atef Zaguia

**Affiliations:** ^1^Department of Electrical and Computer Engineering, North South University, Bashundhara, Dhaka 1229, Bangladesh; ^2^School of Electrical Engineering and Computer Science, Gwangju Institute of Science and Technology, Gwangju 61005, Republic of Korea; ^3^Department of Computer Science, College of Computers and Information Technology, Taif University, Taif 21944, Saudi Arabia

## Abstract

We live in a world where people are suffering from many diseases. Cancer is the most threatening of them all. Among all the variants of cancer, skin cancer is spreading rapidly. It happens because of the abnormal growth of skin cells. The increase in ultraviolet radiation on the Earth's surface is also helping skin cancer spread in every corner of the world. Benign and malignant types are the most common skin cancers people suffer from. People go through expensive and time-consuming treatments to cure skin cancer but yet fail to lower the mortality rate. To reduce the mortality rate, early detection of skin cancer in its incipient phase is helpful. In today's world, deep learning is being used to detect diseases. The convolutional neural network (CNN) helps to find skin cancer through image classification more accurately. This research contains information about many CNN models and a comparison of their working processes for finding the best results. Pretrained models like VGG16, Support Vector Machine (SVM), ResNet50, and self-built models (sequential) are used to analyze the process of CNN models. These models work differently as there are variations in their layer numbers. Depending on their layers and work processes, some models work better than others. An image dataset of benign and malignant data has been taken from Kaggle. In this dataset, there are 6594 images of benign and malignant skin cancer. Using different approaches, we have gained accurate results for VGG16 (93.18%), SVM (83.48%), ResNet50 (84.39%), Sequential_Model_1 (74.24%), Sequential_Model_2 (77.00%), and Sequential_Model_3 (84.09%). This research compares these outcomes based on the model's work process. Our comparison includes model layer numbers, working process, and precision. The VGG16 model has given us the highest accuracy of 93.18%.

## 1. Introduction

According to the World Cancer Research Fund, among all cancers, skin cancer is the 19th most common. People in the USA, Canada, and Australia have been diagnosed at the highest increasing rate over the past few decades. Skin cancer happens due to the uneven development of melanocytic skin cells [1]. Among all skin cancers, malignant and benign are the deadliest. A malignant tumor is a type of cancerous tumor that spreads and expands in a patient's body. They can infiltrate other tissues and organs and develop and spread unchecked. Many malignant skin growths have symptoms that can be identified as precursors. A precursor is a group of aberrant cells that may develop into cancer. Precancerous is another term for a precursor. Some precancerous skin growths have a minimal chance of developing into cancer, whereas others have a very high chance. There are many kinds of malignant skin growth, like melanoma, carcinoma, sarcoma, squamous cell carcinoma, and skin lymphoma [2]. The importance of detecting and treating cancer in early malignant skin growth cannot be overstated [3]. In many cases, complete excision (surgical removal) leads to healthiness. On the contrary, a benign tumor has the capability to develop, but it is not going to spread. When it comes to benign skin growths, knowing the common signs and symptoms of those that could be malignant is critical, as is seeking medical attention when skin growths show suspect. Benign skin growths include seborrheic keratoses, cherry angiomas, dermatofibromas, skin tags (acrochordon), pyrogenic granulomas, and cysts (epidermal inclusions). Here, Figure 1 shows cancer cases in men and women of different ages. Incidence rates rise steadily from around the age of 20 to 24 and more sharply in males from around the age of 55 to 59. Females aged 90 and up had the greatest rates, while males aged 85 to 89 had the lowest. Females have much greater rates of cancer than males in earlier age groups, while females have significantly lower rates of cancer in older age groups. The disparity is greatest between males and females between the ages of 20 and 24, when girls have a 2.5-fold greater age-specific incidence rate than males [4].

There are many deadly diseases in the current world. Skin cancer is one of them. Skin cancer cells grow and spread like tumors in the human body. If left unchecked, this tumor can become deadly by affecting other body tissues and organs. People go through expensive and time-consuming treatments to cure skin cancer but yet fail to lower the mortality rate. Detection of skin cancer at an early stage can help to reduce mortality. Machine Learning (ML) models have come up with the solution. Deep Learning, notably the Convolution Neural Network, can be used to identify skin cancer quickly and cheaply using image classification. It has become a lifesaver for poor people. These ML models are more accurate and faster in terms of detecting skin cancer via image classification. Medical science is developing in today's world. Previously, skin cancer was detected manually, which was difficult and expensive. But due to the advancement of deep learning in the medical science field, it has become much easier. For this reason, the CNN is proposed in the systems of this study to detect skin cancer.

Many researchers have applied CNN architectures to skin cancer datasets to develop a better solution to detect skin cancer at an incipient phase. Using CNN to analyze the skin lesions in dermoscopy images was introduced by the authors of [5]. They achieved an accuracy of 80.3% using deep CNN on the International Skin Imaging Collaboration (ISIC) dataset. A convolutional-deconvolutional architecture is used to segment the data. Another group of researchers worked on the same dataset, but they used CNN based on symptomatic feature extraction [6]. After segmenting the dermoscopic images using the feature extraction approach, the characteristics of the afflicted skin cells are retrieved in this work. They got an accuracy of 89.5%. A paper was published on the vision-based classification of skin cancer. They used CNN and the VGG16 [7]. They worked on three different training systems and got an accuracy of 78%. A deep convolutional neural network, logistic regression, and a fine-tuned, pretrained VGG16 were among the three models used in that system. A region-based CNN with ResNet152 was also applied by a group of researchers on the ISIC dataset of 2742 dermoscopic images, where they got an accuracy of 90.4% [8].

Researchers have worked in many ways with CNN architectures to detect skin cancer. By changing CNN models, layer numbers, and even datasets referred to, their work could not give an accuracy of more than 90.4%. This paper worked with six different convolutional neural models. This research paper clearly distinguishes the accuracy and work method among the six deep learning models. Where other referred papers could not achieve the same result using these models, in our case VGG16 had a 93% accuracy rate, which is the highest among the referred papers. In the VGG16 architecture, the number of parameters is increased in this system. By adding some layers, the number of parameters increased to approximately 134 million. Medical science and deep learning researchers can both benefit from this research project. This research shows differentiation among the models and architectures of deep learning, focusing only on skin cancer. The detailed information gathered through this research can help the next generation of researchers achieve total accuracy in finding skin cancer. The dataset used in this system is large and has dermatoscopic images. This system gave higher accuracy than the referred systems and also has a detailed comparison between the models.

This research shows the comparison between some CNN models based on their work processes. CNNs are one of the most common types of neural networks that have been used for picture recognition and image classification. CNNs are also commonly utilized in domains such as object detection, face recognition, and so on. Through backpropagation, CNN learns to build spatial hierarchies of information automatically and adaptively using many essential elements, such as pooling (mx/average) layers, convolution layers, and fully connected layers [9]. These features help to identify skin cancer better than dermatologists can with their eyes. These features are used to get the best results. A comparison has been made between the received results and various CNN models. The dataset is fully prepared for our model to work on. The convolutional layer is utilized to separate different functionality from input pictures. Pretrained models like SVM, VGG16, and ResNet50 are used, as well as some sequential models with different parameters. This research could work better than the existing systems and help dermatologists around the world.

Section 2 provides the method and methodology of convolutional neural networks, where all the convolutional work processes have been stated. This section also contains information about SVM, VGG16, ResNet50, and sequential models. In Section 3, we have the results and comparison of our models. Finally, our conclusion is provided in Section 4.

## 2. Method and Methodology

For this research, many CNN models have been implemented. As CNN is mostly based on convolutional layers, models with different numbers of layers like SVM, VGG16, ResNet50, and sequential are used. All the models are applied to a single dataset. The dataset is prepared and trained with these models. The work process of these trained models has been distinguished by the accuracy acquired.

### 2.1. Materials and Tools

Running these systems Python as a programming language is used because its library is very large. Libraries like Pandas and Matplotlib are used to show statistical analysis and plot visual graphs. Google Colab has worked as an IDE for these systems. In this research, a core i5 laptop was used as a workstation. Rather than the integrated RAM (8 GB) and graphics (2 GB) of the laptop, Google Colab's integrated RAM and GPU are used. TensorFlow was introduced as a free and open source Python library. TensorFlow is used to do machine learning techniques using dataflow. It also helped train models and compute values. Google Drive helped to store the dataset.

### 2.2. Dataset

A lot of data is needed to work on deep learning studies because ML or AI models cannot be trained without data. In this research, a dataset from Kaggle is used, which is named “‘Skin Cancer' Malignant vs. Benign”. Kaggle is one of the top resources for data scientists and machine learners looking for datasets. This dataset has a total of 6594 images [10]. The dataset is divided into two sections: train (5274 images), which is used to train the models, and test (1320 images), which is used to test the accuracy of the trained models. Both sections have malignant (total of 2994 images) and benign (total of 3600 images) cancer images. The image sizes are (224 × 224). They are all high quality pictures. The ISIC-Archive rights bind all of the data rights for this dataset.

### 2.3. Convolutional Neural Network (CNN)

Neural networks are one of the most beautiful programming paradigms ever devised. Anyone can instruct the computer what to do in the traditional method of programming, breaking large issues down into many small, carefully defined jobs that the computer can readily complete. In a neural network, on the other hand, users do not tell the computer how to solve their problems [11]. Rather, it learns from observational data and comes up with its own solution to the problem. CNN's weight-sharing function, which reduces the number of network parameters that can be trained and helps to avoid overfitting by the model and increase generalization, is one of the key reasons for considering CNN in such a circumstance.

Both the feature extraction and classification layers load data simultaneously in CNN, which makes the model's output more ordered and dependent on the extracted features. Convolutional neural networks rely on three fundamental concepts: pooling, shared weights, and local receptive fields [12].

Figure 2 depicts CNN's fundamental conceptual model, with layers of several kinds explained in the following sections. A CNN-based model is basically built up with a limited number of processing units that master multiple levels of abstraction from incoming data (such as the image in Figure 2). It takes datasets as input. Then it runs multiple layers, like convolutional layers, followed by a pooling layer. At the end, there is a fully connected layer and an output. Between the input and FC layers, there are many hidden layers. The hidden layers study and extract low-level properties, whereas the initiatory elements (with less abstraction) learn and retrieve high-level elements (with higher abstraction) [13].

Figure 3 shows the work process of the system block diagram, which is described below. This system begins by preprocessing data taken from Google Drive into its system. Then data is normalized by null value reduction, image resizing, labeling images, and many more. Normalizing data is one of the most important factors in this project as it helps to decrease value loss. After processing, the data system is trained with six different neural network models (SVM, VGG16, ResNet50, sequential 1/2/3). After training data with trained images, it is fine-tuned to get the maximum accuracy. One of the most important tasks in this process is to check the overfitting and underfitting of these models. When the system is ready for the final process, test data is used to predict and get an accurate output. This work process is maintained throughout the study.

#### 2.3.1. Convolutional Layer

For every CNN architecture, convolutional layers are the most integral feature. It comprises a collection of convolutional kernels (filters) that are highly integrated to build an output feature map from the source data (N-dimensional parameters).  Figure 4 shows how a convolutional network takes data from an input and gives an output.

A single convolutional layer has an input volume. From the input source, it filters out some segments of data, with the activation value reserved for those. Then the activation value is processed and sent to the output activation volume. All the communication is done using kernel tricks. A kernel is an array of continuous or integer values, with every value reflecting the kernel weight. All the kernel weights are allocated random integers when the training process of a CNN model begins (other ways of initializing the weights are also available). The weights are then fine-tuned with each training epoch, and the kernel learns to extract significant information.

#### 2.3.2. Pooling Layer

Feature maps are subsampled using pooling layers (produced following convolution operations), compressing larger feature maps into smaller ones. The most significant features (or content) for each pool stage are always kept when the feature maps are shrunk. Pooling is done in the same way as convolution is done, by determining the operation stride and the size of the region of pooling. In different pooling layers, several types of pooling techniques are utilized, among them are maximum, average, minimum, gated, and tree pooling, to name a few [14]. The most popular and often used pooling approach is max-pooling.

#### 2.3.3. Fully Connected

Fully connected layers, where each cell in one layer is related to every cell in the preceding layer, make up the last component (or layers) of the convolution layer (which is used for classification). The CNN architecture's output unit (classifier) is the final layer of fully connected layers. FC layers (FCLs) are one of many kinds of feedforward artificial neural networks (ANN) that work similarly to a neural network like multilayer perceptron (MLP) [15]. The fully connected layers receive input after the last convolutional or pooling layer in accordance with a set of parameters (feature maps), which are compressed to generate a variable, which is then passed into the FC layer to construct CNN's end result.

#### 2.3.4. Confusion Matrix

A confusion matrix (also known as an error matrix) is a quantitative approach to describing picture categorization accuracy, and it is a table that summarizes the results of a classification model. The number of correct and incorrect estimates is tallied and burned away by class. The confusion matrix is based on true negative (TN), false negative (FN), true positive (TP), and false positive (FP). The confusion matrix (CM) helps to find other results more accurately. Some of the equations used to calculate CM are given below in equations (1) and (2) [16]:

(1) $$\begin{array}{c} {\text{TN}}_{i}\;=\;\sum_{j=1,j\neq 1}^{n}\sum_{k=1,k\neq 1}^{n}a_{ij}, \end{array}$$

(2) $$\begin{array}{c} {\text{FN}}_{i}=\sum_{j=1,j\neq 1}^{n}a_{ij}. \end{array}$$

Figure 5 shows a confusion matrix diagram.

CM has two main points. One is the true label, where all the stored true value is saved. This label is situated on the *x*-axis. Another is the predicted label, where results from the trained systems are given to compare with the original true value. This label is situated on the *y*-axis. From all the values, the true positive part gives the correct result. The true positive part can be found on a graph where values with the same label from both axes (*x* and *y*) are matched. With the help of CM, other equations can be run as stated below.

(3) $$\begin{array}{c} \text{Accuracy}=\frac{\#\text{ of correct predictions}}{\text{total }\#\text{ of predictions}}=\frac{\text{TP}+\text{TN}}{\text{TP}+\text{TN}+\text{FP}+\text{FN}}. \end{array}$$

In equation (3), the accuracy formula is given. Accuracy can be calculated through CM parameters. Here, the total number of correct predictions is divided by the total number of predictions:

(4) $$\begin{array}{c} \text{Precision}=\frac{\text{True Positive}}{\text{True Positive}+\text{False Positive}}. \end{array}$$

In equation (4), the precision formula is given. Precision can also be calculated with CM parameters. Here, the total number of true positive cases is divided by the summation of the number of true positive cases and the number of false positive cases.

### 2.4. Convolutional Neural Network Models

The CNN model handles data in a grid pattern, such as images. It is intended to automatically learn the spatial hierarchies of features. CNN analyzes the raw pixel data from the image, trains the model, and then extracts the features for improved categorization. A number of CNN models like SVM, VGG16, ResNet50, and sequential are presented here that use unstructured growth of skin cancer images as inputs to specify benign and malignant skin cancer.

#### 2.4.1. SVM Model

SVM has three major qualities when used to predict the regression equation. To begin, SVM uses a collection of linear functions specified in a high-dimensional area to calculate the regression. After that, SVM uses a Vapnik-insensitive loss function to evaluate risk and perform regression estimation via risk minimization. Finally, SVM employs a risk function that combines empirical error with a regularization component obtained from the Selectively Reliable Multicast Protocol (SRMP) [17]. For classification problems, SVM works as a supervised learning-based binary classifier that outperforms other classification algorithms [18]. An SVM distinguishes between two classes by creating a classification hyperplane in a high-dimensional feature space [19].

Figure 6 shows the internal architecture of the SVM model, which is described below. The SVM architecture worked with benign and malignant datasets in the simplest way. In this project, SVM used 2 types of layers (M∗M) of CNN for skin cancer detection via image classification. It took input (benign vs. malignant datasets) in the beginning and then sent it to the hidden layers. After a convolutional layer, it passes through a pooling layer. All the segments are connected with all the previous segments. In hidden layers, SVM only passes the weights (*x*, *x*) of image data. Bias is checked regularly and added to the final calculation to reduce loss and increase precision.

#### 2.4.2. VGG16 Model

The 2014 ILSVRC (Imagenet) competition was won by VGG16, a convolutional neural network (CNN) architecture. It is widely recognized as one of the most advanced vision model architectures yet devised. The convolutional and max-pool layers are placed in the very same way throughout the architecture. It finishes with two fully connected layers and a softmax for the outcome [20]. The number 16 in VGG16 reflects the fact that it has 16 layers of varying values. With an estimated 138 million elements, this system is fairly large [21].  Figure 7 shows all the 16 layers of the VGG16 model.

All the 16 layers of the vgg16 model are divided into 5 types of layers (conv, ReLU, max-pooling, softmax, and fully connected). The convolutional layer takes a 224 by 224 RGB value with a fixed length as the source. The data is transformed by a bunch of convolutional layers with a 3 × 3 visual field (the minimum size to retain the concepts of rightmost/leftmost, rise/bottom, and core). The convolutional layer is followed by a max-pooling layer. Convolution and ReLU process the data together. In a few of the configurations, it additionally includes 11 filters of convolution, which is usually regarded as a proportional change of the input networks (followed by nonlinearity). Every convolution stride is specified as a single pixel, and the spatial padding of such a convolution layer source is set the same as a single pixel for 3 by 3 convolution layers, following convolution, keeping spatial resolution. Instead of having a bunch of hyperparameters, VGG16 concentrated on having a 3 × 3 filter input layer with a stride of 1 and would always use the same padding and max-pool structure. Spatial pooling is done via layers of 5 max-pooling that replicate part of the convolutional layers.

#### 2.4.3. ResNet50

ResNet50 is a residual network with 50 layers and 26 million parameters. In 2015, Microsoft introduced the residual network, a deep convolutional neural network model. Rather than learning features, the residual network learns from residuals, which are the subtraction of features learnt before the inputs of the layer. The skip connection was used by ResNet to transport information across layers [22].  Figure 8 shows how all the 50 layers are connected to each other in ResNet50. The architecture of ResNet50 is separated into 4 stages, as seen in the picture given. An impression with a size that is multiples of 32 and a channel width of three can be accepted by the system. For the sake of clarity, we will suppose the filter size is 224 by 224 by 3. For preliminary convolution and max-pooling, each ResNet design employs seventy-seven percent and thirty-three percent kernel sizes, correspondingly. Following that, the network's first step begins, which is made up of three residual blocks, all with all three layers. In all 3 layers of stage 1's unit, the kernels then used to execute the convolution process are 64, 64, and 128 in size, correspondingly.

The curvy arrow indicates the same connection. The dotted connection arrows represent that stride two is used for convolution in the residual block, providing a 1/2 input in terms of height and breadth but twice the channel width. The average pooling layer is the system's bottom layer. Then comes a fully linked layer of a thousand neurons. Malignant (total 2994 images) and benign (total 3600 images) cancer images are included in our dataset.

#### 2.4.4. Sequential Model

The simplest technique for creating a machine learning system with a model is sequential. It allows you to build a model layer by layer. Every layer contains weights that are identical to those of the one above it [24]. It is made up of convolutional and pooling-type sequential layers whose job is to extract patterns from an image.

Figure 9 shows how layers are built in a sequential model. The number of filters in convolutional layers often grows as the network gets deeper, while the number of rows and columns decreases. Like the above structure, a sequential model is built with layers like conv, ReLU, max-pooling, dense, and fully connected. After a convolutional and ReLU layer, there is always a pooling layer conv1-Lu1-maxPool1. The bigger the system gets, the larger the number of parameters. The key benefit of this design is its ease of implementation. But if one wishes to learn more complex patterns, he or she needs a lot of depth, which leads to a vanishing gradient problem. In sequence modeling, a neural network takes in a unique set of datasets and generates a vast variety of outputs.

## 3. Result and Analysis

This system has been run on Google Colab with the help of the Python 3 Google compute engine backend GPU and shared RAM (12.69 GB). The dataset was uploaded to Google Drive for easy use on Google Colab. Six systems have been run in six different Colab files to compare convolutional neural network models. All the systems worked successfully and gave us the expected results, which are discussed in this section.

### 3.1. SVM

In this system, the image dataset is normalized. Then the dataset is fit with training data and then predicted with test data.  Figure 10 shows the training and test data with benign and malignant pictures.

The above graph shows the data of benign and malignant images that were taken from Kaggle. Here, the graph is divided into two sections: train (a) (2637 images), which is used to train the models, and test (b) (660 images), which is used to get the accuracy of the trained models. In the training graph, benign images are 1440 in number and malignant images are 1197 in number. In the test graph, benign images are 360 in number and malignant images are 300 in number. Both sections have malignant (total 2994 of images) and benign (total of 3600 images) cancer images.

In Figure 11, pictures of malignant and benign skin cancer were shown separately with tags. All the pictures are resized to 244 ∗ 244 in Figure 10. Here are two rows and 5 columns of predicted malignant and benign images. These images are sent through the trained SVM model. From the 10 picture predictions, the system gave six benign images and four malignant images.

Figure 12 shows the confusion matrix SVM model. The confusion matrix shows the predicted result based on test images on the SVM system. The confusion matrix has a true label on the *y*-axis and a predicted label on the *x*-axis. True labels show the true result of a predicted image result, and a predicted label shows only the predicted image result, which can be true or false. These results are then cross-checked with the true results. Here we got 66 and 43 images of benign and malignant predictions, respectively.

This system provided a predicted accuracy of 83.48% as this was a simple classification model.

### 3.2. VGG16

Figure 13 shows the accuracy and loss function graph of the VGG16 model. There are two curves in each graph. One is the train curve and the other is the test curve. The training curve is always higher in model accuracy (a) than the test curve due to overfitting or training the model on a particular dataset. In test loss (b), it gives the value of 0.2603 and in test loss it gives the value of 0.1716 at the highest accuracy of 93.18%.

Table 1 shows the parameter values used in this system. All the 16 layers of the VGG16 model create some parameters. The number of parameters increases as the layers go deep. The 1st convolutional layer has 1792 parameters, whereas convolutional 1 in block 5 has a parameter of 2359808. The 13 convolutional layers are divided into 5 blocks. Each block ended with a max-pooling layer. The max-pool layer did not create any parameters. In every layer, a number of parameters are created because changes are made to the output shape of the data. The maximum number of parameters is created on the last two fully connected layers. The total number of parameters of this VGG16 system is 134,264,641. All are trainable parameters.

Table 1 shows all the layers and the total number of parameters of our model (VGG16).

Table 2 shows the highest accuracy secured by this model (VGG16) with train loss and test loss at peak result. Data for the total parameters and layers of this system is also shown. Train loss and test loss results come from an in-built loss function of the system. It helped the system track data loss and recover it. After training and applying a test image set, the VGG16 system gave us a train loss of 0.2603 and a test loss of 0.1716, calculated on the loss function. These values are collected from the epoch of highest accuracy. The highest accuracy of this system is 93.18%.

### 3.3. ResNet50

Figure 14 shows the accuracy and loss function graph of the ResNet50 model. There are two curves in each graph. One is the train curve, and the other is the test curve. Though Figure 14 shows that the balance between test and train curves in model accuracy (a) is slightly different, the balance is quite good in the model loss (b) graph. The accuracy measurement is set at 100 percent where the number of epochs is set at 30. The best result one can get from a system is defined by the test curve in model accuracy and the lower test curve for model loss graph. In test loss, it gives a value of 0.2359 and in test loss 0.4305 at the highest accuracy of 84.39%.

Table 3 shows all the layers and the total number of parameters of our model (ResNet50). Here, with the built-in 50 layers of ResNet, we also added 10 more layers for better accuracy. Convolutional and pooling layers are added. As a result, the total number of parameters is increased from the actual number of parameters of the ResNet50 model. The actual number of parameters of ResNet50 is around 23.5 million, which means we get a new total number of parameters of around 25 million. Among 25 million parameters, 53,120 come out as nontrainable. As the value is too small compared to the trainable number of parameters, it did not bother much.

Table 4 shows the highest accuracy secured by this model (ResNet50) with train loss and test loss at peak result. Data for the total parameters and layers of this system is also shown. Train loss and test loss results come from an in-built loss function of the system. It helped the system track data loss and recover it. After training and applying a test image set, the ResNet50 system gave us a train loss of 0.2359 and a test loss of 0.4305, calculated on the loss function. These values are collected from the epoch of highest accuracy. The highest accuracy of this system is 84.39%.

### 3.4. Sequential Model 1

Figure 15 shows the accuracy and loss function graph of the sequential model 1. It is one of the three systems built on a sequential model. In this system, fewer parameters are used than in the other two systems. There are two curves in each graph. One is the train curve, and the other is the test curve. Though it shows that the balance between test and train curves in model accuracy is slightly different, the balance is quite good in the model loss graph. The accuracy measurement is set at 100 percent where the number of epochs is set at 30. The higher the test curve in model accuracy (a) and the lower the test curve in the model loss (b) graph, the better the result one can get from a system. In test loss, it gives a value of 0.4578 and in test loss it is 0.5695 at the highest accuracy of 74.24%.

Figure 15 shows the accuracy and loss function graph of the sequential model 1. It is one of the three systems built on a sequential model. In this system, fewer parameters are used than in the other two systems. There are two curves in each graph. One is the train curve, and the other is the test curve. Though it shows that the balance between test and train curves in model accuracy is slightly different, the balance is quite good in the model loss graph. The measurement of accuracy is set to 100 percent, and the number of epochs is set to 30. The best result one can get from a system is represented by the test curve in model accuracy (a) and the test curve in model loss (b) graph. At test loss, it gives a value of 0.4578 and at test loss it is 0.5695 at the highest accuracy of 74.24%.

Table 5 shows all the layers and the total number of parameters of our model (sequential model 1). Here, a system is built with 15 layers for better accuracy. Convolutional and pooling layers are added. As a result, the total number of parameters has increased. The sequential model 1 is built with 15 layers as shown in Table 5. The highest number of parameters created on a dense layer is 13,52,100. The total number of parameters in this system is around 1.3 million. Among 1.3 million parameters, nothing comes out as nontrainable. As all the parameters are trainable, the best accuracy from this model is acquired.

Table 6 shows the highest accuracy secured by this model (sequential model 1) with train loss and test loss at peak result. Data for the total parameters and layers of this system is also shown. Train loss and test loss results come from an in-built loss function of the system. It helped the system track data loss and recover it. As the number of parameters for this system is lower than the others, this model did not give much accuracy. The test loss value was also greater than the train loss function. That is why parameters were increased in the next systems to observe the changes in accuracy with the change of the systems parameters. After training and applying a test image set, the sequential model 1 system gave us a train loss of 0.4578 and a test loss of 0.5695, calculated on the loss function. These values are collected from the epoch of highest accuracy. The highest accuracy on this system is 74.24%.

### 3.5. Sequential Model 2

Figure 16 shows the model accuracy and model loss graph of the sequential model 2. It is one of the three systems built on a sequential model. In this system, fewer parameters are used than in the other two systems. There are two curves in each graph. One is the train curve, and the other is the test curve. Though it shows that the balance between test and train curves in model accuracy is slightly different, the balance is quite good in the model loss graph. The accuracy measurement is set to 100 percent, and the number of epochs is set to 30. The best result one can get from a system is represented by the test curve in model accuracy (a) and the test curve in model loss (b) graph. At test loss, it gives a value of 0.4249 and at test loss it is 0.4549 at the highest accuracy of 77.00%.

Table 7 shows all the layers and the total number of parameters of our model (sequential model 2). Here, a system is built with 15 layers for better accuracy. Convolutional and pooling layers are added. As a result, the total number of parameters has increased. The sequential model 2 is built with 13 layers as shown in Table 7. The highest number of parameters created on a dense layer is 1730688. The total number of parameters in this system is around 1.7 million. Among 1.7 million parameters, nothing comes out as nontrainable. As all the parameters are trainable, the best accuracy from this model is acquired.

Table 8 shows the highest accuracy secured by this model (sequential model 2) with train loss and test loss at peak result. Data for the total parameters and layers of this system is also shown. Train loss and test loss results come from an in-built loss function of the system. It helped the system track data loss and recover it. As the number of parameters for this system is lower than the others, this model did not give much accuracy (<80%). The test loss value was also greater than the train loss function. That is why parameters were increased in the next system to observe the changes in accuracy with the change of the system parameters. After training and applying a test image set, the sequential model 2 system gave us a train loss of 0.4249 and a test loss of 0.4549, calculated on the loss function. These values are collected from the epoch of highest accuracy. The highest accuracy on this system is 77.00%.

### 3.6. Sequential Model 3

Figure 17 shows the accuracy and loss function graph of the sequential model 3. It is one of the three systems built on a sequential model. In this system, a larger number of parameters are used than in the other two systems. There are two curves in each graph. One is the train curve, and the other is the test curve. Though it shows that the balance between test and train curves in model accuracy (a) is slightly different, the balance is quite good in the model loss (b) graph. The accuracy measurement is set to 100 percent, and the number of epochs is set to 30. The best result one can get from a system is defined by the test curve for model accuracy and the lower test curve for model loss graph. At test loss, it gives a value of 0.1535 and at test loss it is 0.4235 at the highest accuracy of 84.09%.

Table 9 shows all the layers and the total number of parameters of our model (sequential model 3). Here, this system is built with 13 layers for better accuracy. Convolutional and pooling layers are added. As a result, the total number of parameters has increased. The sequential model 2 is built with 13 layers as shown in Table 9. The highest number of parameters created on a dense layer is 5537920. The total number of parameters in this system is around 5.6 million. Among 5.6 million parameters, 384 come out as nontrainable. As the value is too small compared to the trainable number of parameters, it did not bother much.

Table 10 shows the highest accuracy secured by this model (sequential model 3) with train loss and test loss at peak result. Data for the total parameters and layers of this system is also shown. Train loss and test loss results come from an in-built loss function of the system. It helped the system track data loss and recover it. As the number of parameters of this system is greater than the others, this model gave us much better accuracy (>80%). The test loss value was also greater than the train loss function. That is why parameters were increased in this system to observe the changes in accuracy with the change of the system's parameters. After training and applying a test image set, the sequential model 3 system gave us a train loss of 0.1535 and a test loss of 0.4235, calculated on the loss function. These values are collected from the epoch of highest accuracy. The highest accuracy on this system is 84.09%.

### 3.7. Comparison between Models

Table 11 gives us the overall observation of all of the six systems of convolutional neural network models introduced in this research. We have used models with different numbers of layers, like VGG16 (16 layers), sequential model 3 (13 layers), and others. We also increased the number of parameters from 1.3 million to 134.2 million. We also noted the train loss and test loss of data at the peak accuracy of these systems. The accuracy changed for different numbers of parameters and different numbers of layers. Changes in the number of layers brought changes in accuracy. We can see that ResNet50 with 60 layers gave greater accuracy than sequential models with a lower number of layers. The great finding from this research is that the increase in the number of parameters increases precision. The decrease in the test loss value also increased the accuracy of the system. From this table, we can observe that sequential model 1 has the lowest number of parameters (1,371,241) and the highest value of the test loss (0.5696) function. As a result, it has given a low accuracy (74.24%). On the contrary, the VGG16 model has the highest number of parameters (134,264,6641) and the lowest value of the test loss (0.1716) function. As a result, it has given the highest accuracy (93.18%) among the systems.

In Table 12, it is clear that this system achieved the highest accuracy. Many convolutional neural network models have been used, and many paths and instructions have been followed to detect skin cancer via image classification. To help dermatologists detect skin cancer more effectively, the VGG16 system described in this paper will work more accurately.

## 4. Conclusion

There are many deadly diseases in the current world. Skin cancer is one of them. The best way is to diagnose it as early as possible. Medical science has developed in today's world. Previously, skin cancer was detected manually, which was difficult and expensive. But due to the advancement of deep learning in the medical science field, it has become much easier. Deep Learning, specifically CNN, can be used to rapidly detect skin cancer, which is easy and less expensive. For this reason, the CNN is proposed in this study to detect skin cancer. In this research, we used a variety of convolutional neural network models (SVM, VGG16, ResNet50, sequential model 1, sequential model 2, and sequential model 3).

After applying different convolutional models to the dataset, an accuracy of 83.48% from SVM, 84.39% from ResNet50, 93.18% from VGG16, 74.24% from sequential model 1, 77.00% from sequential model 2, and 84.09% from sequential model 3 was acquired. The best results from this research come from the VGG16 model. This system was built to detect skin cancer. This will help doctors detect skin cancer easily and quickly.

In the future, more advanced convolutional neural network models for this comparison can be added. The information regarding deep learning models on skin cancer gathered in this research paper can help the next generation of researchers achieve 100% accuracy in detecting skin cancer. As this research paper is only based on two types of skin cancer, research can be done on other types of skin cancer using the same methods. These systems can apply to large datasets. It will help to find more accurate models for skin cancer detection via image classification.

## Figures and Tables

**Figure 1:** Melanoma skin cancer incidence by age [4].

**Figure 2:** Conceptual model of CNN.

**Figure 3:** Systems block diagram.

**Figure 4:** One convolutional layer [13].

**Figure 5:** Confusion matrix diagram.

**Figure 6:** SVM architecture.

**Figure 7:** Basic architecture of VGG16 model.

**Figure 8:** ResNet50 model architecture [23].

**Figure 9:** Architecture of conventional sequential model [25].

**Figure 10:** Train and test data visualization. (a) Train data visualization. (b) Test data visualization.

**Figure 11:** Images of malignant and benign skin cancer.

**Figure 12:** Confusion matrix of SVM model.

**Figure 13:** Accuracy and loss graph of VGG16. (a) Model accuracy. (b) Model loss.

**Figure 14:** Accuracy and loss graph of ResNet50. (a) Model accuracy. (b) Model loss.

**Figure 15:** Accuracy and loss graph of sequential model 1. (a) Model accuracy. (b) Model loss.

**Figure 16:** Accuracy and loss graph of sequential model 2. (a) Model accuracy. (b) Model loss.

**Figure 17:** Accuracy and loss graph of sequential model 3. (a) Model accuracy. (b) Model loss.

**Table 1:** Layers and parameters of VGG16.

VGG16 model		
Type of layers	Outcome structure	Number of parameters
Conv1 (b1)	(Nil, 224 × 224 × 64)	1,792
Conv2 (b1)	(Nil, 224 × 224 × 64)	36,928
Pooling (max)	(Nil, 112 × 112 × 64)	Null
Conv1 (b2)	(Nil, 112 × 112 × 128)	73,856
Conv2 (b2)	(Nil, 112 × 112 × 128)	147,584
Pooling (max)	(Nil, 56 × 56 × 128)	Null
Conv1 (b3)	(Nil, 56 × 56 × 256)	295,168
Conv2 (b3)	(Nil, 56 × 56 × 256)	590,080
Conv3 (b3)	(Nil, 56 × 56 × 256)	590,080
Pooling (max)	(Nil, 28 × 28 × 256)	Null
Conv1 (b4)	(Nil, 28 × 28 × 512)	1,180,160
Conv2 (b4)	(Nil, 28 × 28 × 512)	2,359,808
Conv3 (b4)	(Nil, 28 × 28 × 512)	2,359,808
Pooling (max)	(Nil, 14 × 14 × 512)	Null
Conv1 (b5)	(Nil, 14 × 14 × 512)	2,359,808
Conv2 (b5)	(Nil, 14 × 14 × 512)	2,359,808
Conv3 (b5)	(Nil, 14 × 14 × 512)	2,359,808
Pooling (max)	(Nil, 7 × 7 × 512)	Null
Layer flatten	(Nil, 25088)	Null
Fully connected 1-dense	(Nil, 4096)	102,764,544
Fully connected 2-dense	(Nil, 4096)	16,781,312
Layer dropout	(Nil, 4096)	Null
Layer dense	(Nil, 1)	4097
Total number of parameters: 134,264,641; number of trainable		
parameters: 134,264,641; nontrainable params: null		

**Table 2:** Summary of the analysis of VGG16.

Layer numbers	Parameters	Train loss	Test loss	Highest accuracy (%)
16	134,264,641	0.2603	0.1716	93.18

**Table 3:** Layers and parameters of ResNet50.

Type of layers	Outcome structure	Number of parameters
Functional ResNet50	(Nil, 7 × 7 × 2048)	23587712
Conv_2 (2d)	(Nil, 5 × 5 × 64)	1179712
Conv_3 (2d)	(Nil, 3 × 3 × 64)	36928
Pooling (max)	(Nil, 1 × 1 × 64)	Null
Layer flatten	(Nil, 64)	Null
module_wrapper_8	(Nil, 512)	33280
module_wrapper_9	(Nil, 256)	131328
module_wrapper_10	(Nil, 128)	32896
module_wrapper_11	(Nil, 64)	8256
module_wrapper_12	(Nil, 32)	2080
module_wrapper_13	(Nil, 16)	528
module_wrapper_14	(Nil, 8)	136
module_wrapper_15	(Nil, 2)	18
Total number of parameters: 25,012,074; trainable parameters:		
24,959,274; nontrainable parameters: 53,120		

**Table 4:** Summary of the analysis of ResNet50.

Layer numbers	Parameters	Train loss	Test loss	Highest accuracy (%)
60	24,959,754	0.2359	0.4305	84.39

**Table 5:** Layers and parameters of sequential model 1.

Type of layers	Outcome structure	Number of parameters
Conv-1 (2d)	(Nil, 222 × 222 × 50)	1400
Pooling-1 (max)	(Nil, 111 × 111 × 50)	Null
Layer Dropout-1	(Nil, 111 × 111 × 50)	Null
Conv_2 (2d)	(Nil, 109 × 109 × 20)	9020
Pooling-2 (max)	(Nil, 54 × 54 × 20)	Null
Layer Dropout-2	(Nil, 54 × 54 × 20)	Null
Conv_3 (2d)	(Nil, 54 × 54 × 20)	3620
Pooling-3 (max)	(Nil, 26 × 26 × 20)	Null
Layer Dropout-3	(Nil, 26 × 26 × 20)	Null
Layer flatten	(Nil, 13520)	Null
Layer dense	(Nil, 100)	1352100
Layer dropout-4	(Nil, 100)	Null
Layer dense-1	(Nil, 50)	5050
Layer dropout-5	(Nil, 50)	Null
Layer dense-2	(Nil, 1)	51
Total number of parameters: 1,371,241;		
number of trainable parameters: 1,37,241;		
number of nontrainable parameters: null		

**Table 6:** Summary of the analysis of sequential model 1.

Layer numbers	Parameters	Train loss	Test loss	Highest accuracy (%)
15	1,371,241	0.4578	0.5695	74.24

**Table 7:** Layers and parameters of sequential model 2.

Type of layers	Outcome structure	Number of parameters
Conv-1 (2d)	(Nil, 222 × 222 × 20)	560
Pooling-1 (max)	(Nil, 111 × 111 × 20)	Null
Layer dropout-1	(Nil, 111 × 111 × 20)	Null
Conv-2 (2d)	(Nil, 109 × 109 × 20)	3620
Pooling-2 (max)	(Nil, 54 × 54 × 20)	Null
Layer dropout-2	(Nil, 54 × 54 × 20)	Null
Conv-3 (2d)	(Nil, 52 × 52 × 20)	3620
Pooling-3 (max)	(Nil, 26 × 26 × 20)	Null
Layer dropout-3	(Nil, 26 × 26 × 20)	Null
Layer flatten-1	(Nil, 13520)	Null
Layer dense-1	(Nil, 128)	1730688
Layer dense-2	(Nil, 128)	16512
Layer dense-3	(Nil, 1)	129
Total number of parameters: 1,755,129;		
number of trainable parameters: 1,755,129;		
number of nontrainable parameters: null		

**Table 8:** Summary of the analysis of sequential model 2.

Layer numbers	Parameters	Train loss	Test loss	Highest accuracy (%)
13	1,755,129	0.4249	0.4549	77.00

**Table 9:** Layers and parameters of sequential model 3.

Type of layers	Outcome structure	Number of parameters
Conv-1 (2d)	(Nil, 222 × 222 × 64)	1792
Pooling-1 (max)	(Nil, 111 × 111 × 64)	Null
Normalization-1 batch	(Nil, 111 × 111 × 64)	256
Layer dropout-1	(Nil, 111 × 111 × 64)	Null
Conv-2 (2d)	(Nil, 109 × 109 × 64)	36928
Pooling-2 (max)	(Nil, 52 × 52 × 64)	Null
Conv-3 (2d)	(Nil, 52 × 52 × 64)	36928
Pooling-3 (max)	(Nil, 26 × 26 × 64)	Null
Layer flatten-1	(Nil, 43264)	Null
Layer dense-1	(Nil, 128)	5537920
Normalization-2 batch	(Nil, 128)	512
Layer dropout-2	(Nil, 128)	Null
Layer dense-2	(Nil, 1)	129

Total number of parameters: 5,614,465; number of trainable parameters: 5,614,082; number of nontrainable parameters: 384		

**Table 10:** Summary of the analysis of sequential model 3.

Layer numbers	Parameters	Train loss	Test loss	Highest accuracy (%)
13	5,614,465	0.1535	0.4235	84.09

**Table 11:** A comparative analysis among convolutional neural network models.

Model name	Layer numbers	Parameters	Train loss	Test loss	Highest accuracy (%)	Best accuracy among models (%)
SVM	2				83.48	93.18
Sequential 1	15	1,371,241	0.4578	0.5695	74.24	
Sequential 2	13	1,755,129	0.4249	0.4549	77.00	
Sequential 3	13	5,614,465	0.1535	0.4235	84.09	
ResNet50	60	24,959,754	0.2359	0.4305	84.39	
VGG16	16	134,264,641	0.2603	0.1716	93.18	

**Table 12:** A comparative analysis of relative works.

Research paper	Dataset	NN models	Descriptions	Accuracy (%)
Vision-based skin cancer detection using deep learning	ISIC	VGG16 sequential	Worked on 3 different CNN models	78
Skin cancer detection using CNN	ISIC	Convolutional NN	Used CNN classifier for feature extraction	89.5
Analyzing skin lesions using CNN	ISIC	ResNet50 deep TL	Data balanced was done using data augmentation	80.3
Melanoma diagnosis using deep learning	2742 dermoscopic images (ISIC)	ResNet152 Rb CNN	Specified by mask and Rb CNN, classification was done by ResNet	90.4
Skin cancer detection using CNN (this research)	Kaggle (ISIC)	SVM, VGG16, ResNet50, sequential	Model comparison was done by work process and layers	93.18

## Data Availability

The data utilized to support this research findings are accessible online at https://www.kaggle.com/fanconic/skin-cancer-malignant-vs-benign.
